# ER-α36 mediates cisplatin resistance in breast cancer cells through EGFR/HER-2/ERK signaling pathway

**DOI:** 10.1186/s13046-018-0798-z

**Published:** 2018-06-25

**Authors:** Linlin Zhu, Jiao Zou, Yuanyin Zhao, Xiaomei Jiang, Yang Wang, Xiangwei Wang, Bin Chen

**Affiliations:** 1 Department of Biochemistry and Molecular Biology, Third Military Medical University, Chongqing, 400038 China; 2 Department of Clinical Laboratory, Institute of Surgery Research, Daping Hospital, Third Military Medical University, Chongqing, 400038 China; 3 Department of Urology, Shenzhen University General Hospital, Shenzhen, 518060 Guangdong China

**Keywords:** ER-α36, Cisplatin resistance, Breast cancer, EGFR, HER-2

## Abstract

**Background:**

ER-α36, a novel ER-α66 variant, has been demonstrated to promote tamoxifen resistance in breast cancer cells. However, the role and mechanisms of ER-α36 in cisplatin resistance of breast cancer cells remain unclear. This study investigates the expression and role of ER-α36 in cisplatin resistance of breast cancer cells and elucidates its underlying mechanisms.

**Methods:**

The expression of ER-α36 and the proteins involved in nongenomic estrogen signaling was evaluated by western blot analysis. Cisplatin sensitivity was explored by CCK-8 assay, monolayer colony formation assay and apoptosis assays, respectively. ER-α36 siRNAs/shRNAs and overexpression vector were transfected into cells to down-regulate or up-regulate ER-α36 expression. Loss-and gain-of function assays were performed to investigate the role of ER-α36 in cisplatin sensitivity. The interaction between ER-α36 and EGFR/HER-2 were detected using CoIP. A mouse xenograft model of breast cancer was established to verify the role of ER-α36 in vivo.

**Results:**

ER-α36 is expressed at higher levels in cisplatin-resistant breast cancer cells compared to cisplatin sensitive cells. Cisplatin induced up-regulation of ER-α36 in a dose-dependent manner in breast cancer cells. Overexpression of ER-α36 leaded to cell resistant to cisplatin and knockdown of ER-α36 in cisplatin-resistant breast cancer cells restored cisplatin sensitivity. The up-regulation of ER-α36 resulted in increased activation of nongenomic estrogen signaling, which was responsible for cisplatin resistance. Disruption of ER-α36-mediated nongenomic estrogen signaling with kinase inhibitors significantly inhibited cisplatin-induced expression of ER-α36 and increased cisplatin sensitivity. The in vivo experiment also confirmed that up-regulation of ER-α36 attenuated cisplatin sensitivity in a mouse xenograft model of breast cancer.

**Conclusions:**

The results for the first time demonstrated that ER-α36 mediates cisplatin resistance in breast cancer cells through nongenomic estrogen signaling, suggesting that ER-α36 may serve as a novel target for cisplatin resistance and a potential indicator of cisplatin sensitivity in breast cancer treatment.

## Background

Cisplatin (DDP) is the first generation of platinum drugs [1, 2]. As a cell cycle nonspecific drug, cisplatin is widely used in the treatment of a broad array of solid malignancies, including bladder cancer, lung cancer, ovarian, and breast cancer [3–5]. Cisplatin exerts anticancer effects mainly via the generation of DNA lesions followed by the activation of the DNA damage response and the induction of cancer cell death [4, 6, 7]. Although patients with breast cancer usually have good initial response to cisplatin-based chemotherapy, cisplatin resistance often occurs in clinical practice. Previous studies have shown that activated EGFR/HER-2 signaling and its downstream signaling MAPK/ERK are associated with cisplatin resistance [4]. Recent studies have demonstrated that RAD50 [8] and Pit-1 [9] sensitize human breast cancer cells to cisplatin therapy. At present, the well known molecular mechanisms of cisplatin resistance include increased DNA repair, altered drug cellular accumulation, increased drug cytosolic inactivation, and others [10]. However, the detail mechanisms of cisplatin resistance remain to be elucidated. Searching and developing new therapeutic strategies for overcoming cisplatin resistance is urgently needed to improve the quality of life and patient survival.

ER-α36 (Estrogen receptor-alpha36), a member of ER superfamily with molecular weight 36 kDa, is a recently identified ER-α66 variant [11]. ER-α36 is responsible for estrogen-stimulated cell proliferation and development of ER-positive breast cancer [12]. A large amount of studies have reported that high-level expression of ER-α36 is closely related to tamoxifen resistance in breast cancer cells and is one of the underlying mechanisms of tamoxifen resistance [13–15]. In breast cancer cells overexpressing ER-α36, tamoxifen displays estrogen-like effects and activates MAPK/ERK signaling mediated by ER-α36, which is also known as ER-α36-mediated nongenomic estrogen signaling, and thereby stimulates cell survival and proliferation [16–18]. Recent studies have shown the existence of the ER-α36-EGFR/HER-2 positive regulatory loops in either ER-α negative or ER-α positive breast cancer cells [19, 20]. ER-α36 can physically interact with the EGFR/HER-2. EGFR signaling can activate ER-α36 transcription through an AP1 site in the ER-α36 promoter, and ER-α36 expression stabilizes EGFR protein or positively regulates HER-2 expression [20, 21]. In tamoxifen-resistant MCF-7 cells (MCF-7/TAM), tamoxifen induces expression of ER-α36-EGFR/HER-2 positive regulatory loops and the destruction of the loops restores tamoxifen sensitivity [19]. The role of ER-α36-mediated nongenomic estrogen signaling in tamoxifen resistance has attracted considerable attention, however, the significance of ER-α36 in cisplatin resistance in breast cancer cells has not been investigated.

In our present study, we found that cisplatin induces expression of ER-α36 in a dose-dependent manner in breast cancer cells. The up-regulation of ER-α36 promotes increased activation of ER-α36-mediated nongenomic estrogen signaling, which finally resulted in the generation of cisplatin resistance. Blocking ER-α36 expression or the activity of EGFR/HER-2 or their downstream signaling MAPK/ERK significantly increases cisplatin sensitivity in breast cancer cells. Taken together, these results for the first time reveal that ER-a36 promotes cisplatin resistance in breast cancer cells through nongenomic estrogen signaling, suggesting that targeting ER-α36 may serve as a novel target for cisplatin resistance and a potential indicator of cisplatin sensitivity in breast cancer treatment. Our research provides a novel insight for improving the therapeutic effect of cisplatin, which may be beneficial to the further clinical application of cisplatin in breast cancer treatment.

## Methods

### Cell culture

Human breast cancer cell lines MCF-7, BT474, and MDA-MD-231 were purchased from American Type Culture Collection (ATCC), and characterized by DNA profiling. These original cells were cultured in high-glucose DMEM (Gibco, USA) with 10% FBS (Gibco, USA), in a humid incubator with 5% CO_2_ at 37 °C. MCF-7/DDP cells are 5 μg/mL cisplatin-resistant strains, which were established by culturing MCF-7 with high cisplatin concentrations. Cisplatin was added twice a week after reseeding. Every 2 months, cell survival was analyzed by MTT assay. The IC50 value of cisplatin against MCF-7 and MCF-7/DDP were 4 μg/mL and 15 μg/mL, respectively. MCF-7/DDP cells were four times as resistant to the cytotoxic effect of cisplatin as compared with the initial MCF-7 cells. MCF-7 cells overexpressing ER-α36, MCF-7/ER-α36, and the control cells established as described below were cultured in DMEM medium containing 100 μg/mL G418 (Sigma-Aldrich, St Louis, MO, USA).

### Plasmid preparation and establishment of ER-α36 stable expression or knockdown cell lines

The coding sequence of ER-α36 cDNA was successfully cloned and an ER-α36 expression vector driven by the cytomegalovirus (CMV) promoter was constructed, according to the method established by Wang et al. [22]. MCF-7 cells were transfected with either empty vector or recombinant vector, using Lipofectamine 3000 (Invitrogen, Grand Island, NY, USA) according to the manufacturer’s instructions. After transfection for 72 h, 500 μg/mL G418 was then added to culture medium for stable clone selection. MCF-7 cells stably overexpressing ER-α36 amplified from a single clone were identified by western blot, and then used for the experiments. ER-α36 shRNA lentiviral expression vector (pLVX-shRNA2-Puro-hER-α36, Lenti-shER-α36) and its control vector (pLVX-shRNA2-Puro, Lenti-shNC) were constructed by GenePharma (Shanghai, China). The ER-α36 shRNA target sequences are 5’-ACAUCAUCUCGGUUCCGCA-3’. MCF-7/DDP and MCF-7/ER-α36 cells were plated in six-well plates (5 × 10^5^ cells/well) and were cultured to 60% confluence. Appropriate volumes of lentiviruses were then added according to the multiplicity of infection values recommended by the manufacture. MCF-7/DDP cells expressing ER-α36 shRNA and MCF-7/ER-α36 cells expressing ER-α36 shRNA were selected with 5 μg/mL puromycin and identified by western blot.

### Cell proliferation assay

The cell proliferation was assayed by Cell Counting 8 kit (CCK-8) (Dojindo laboratories, Kumamoto, Japan). The cells were seeded in triplicate into 96-well plates for 12 h and given different treatments for the indicated time; followed by the addition of 10 μL CCK-8 reagents to each well. After incubation at 37 °C for 1 h, the value at OD450 nm was determined according to the manufacturer’s instructions.

### Monolayer colony formation assay

Five hundred cells were seeded in triplicate onto 6-well plates and incubated in medium containing 5 μg/mL cisplatin or equivalent DMSO (vehicle) (Sigma, USA). Every 3–5 days the medium was replaced with fresh medium. After 2 weeks, the colonies were fixed with 100% methanol, stained with 0.1% crystal violet and washed with phosphate buffer solution (PBS). Visible colonies were then counted for quantification.

### Western blot analysis

Isolation of cell extracts and western blot analysis were described previously [23]. The protein concentrations were measured by a BCA protein assay kit (Beyotime Biotechnology, Shanghai, China). Immuno-detection was carried out using ER-α36 (Cell Applications, San Diego, CA, USA), p-ERK1/2 (Cell Signaling Technology, Boston, MA, USA) and total-ERK1/2 (Cell Signaling Technology, Boston, MA, USA), p-EGFR (Cell Signaling Technology, Boston, MA, USA) and total-EGFR (Cell Signaling Technology, Boston, MA, USA), p-HER-2 (Cell Signaling Technology, Boston, MA, USA) and total-HER-2 (Cell Signaling Technology, Boston, MA, USA) antibodies or Tubulin antibody. Tubulin (Beyotime, Shanghai, China) was used as a control for equal loading and transfer.

### Hoechst staining

The cells were seeded in 6-well plates for 12 h and given different treatments for the indicated time. Then the cells were stained with Hoechst 33258 (Beyotime, Shanghai, China) at 10 μg/mL for 10 min in the dark at room temperature and washed 3 times with PBS and photographed under a fluorescence microscope.

### Flow cytometry

Breast cancer cells were harvested and incubated with annexin V-FITC and PI according to the manufacturer’s instructions (BD, 561012), and then the apoptosis was analyzed by a flow cytometer.

### Si-RNA assay

The ER-α36 siRNA target sequences are 5’-GCTAGAGATCCTGATGATTGG-3’. MCF-7/DDP and MCF-7/ER-α36 cells were separately cultured overnight, and then siRNA for ER-α36 (siER-α36) or control siRNA (siNC) was transfected into the cells using lipofectamine 3000 according to the manufacturer’s instructions. Subsequently, the cells were treated with or without 5 μg/mL cisplatin for 48 h, then harvested and used for western blot analysis or cell proliferation assays.

### Co-immunoprecipitation (Co-IP) analysis

Isolation of cell extracts were described previously [23]. Cell lysates were incubated with anti-HER-2 or anti-EGFR antibodies or IgG for 1 h at 4 °C. Then the Protein A/G plus-agarose (Santa Cruz Biotechnology, Dallas, TX, USA) was added and incubated for overnight at 4 °C. The precipitates were then extensively washed with the PBS, re-suspended in loading buffer, separated on SDS-polyacrylamide gel electrophoresis and probed with anti-ER-α36 antibody as described before [23].

### Animal experiments

Five-week-old female nude mice were purchased from the Laboratory Animal Center of China (Shanghai, China). The mice were randomized into 2 groups with 10 mice per group and then separately inoculated subcutaneously MCF-7/ER-α36 and MCF7/V cell suspension. Every mouse was inoculated 1 × 10^7^ cells suspending in 0.1 mL PBS. When palpable tumors formed, every group were randomly divided into two groups, and either treated with DMSO (control), or cisplatin (4 mg/kg) by intraperitoneal injections every other day for 2 weeks, respectively. After that, the mice were sacrificed and the xenograft tumors were harvested. The volumes were estimated using the following formula: volume = width^2^ × length × 1/2. Tumor tissues were processed for ER-α36 expression analysis.

### Statistical analysis

The data were expressed as the mean ± SD unless otherwise stated. Statistical comparisons between groups were performed by one-way analysis of variance (ANOVA), followed by student’s *t*-test. *P* < 0.05 was considered significant.

## Results

### Cisplatin induces up-regulation of ER-α36 in breast cancer cells

MCF-7/DDP cells were found to be resistant to 5 μg/mL cisplatin, compared with the wild-type MCF-7 cells, as shown in Fig. 1a and b. Meanwhile, ER-α36 expression was significantly higher in MCF-7/DDP cells than in MCF-7 cells (Fig. 1c and d), indicating that cisplatin may induce ER-α36 expression in the process of cisplatin resistance formation. Corresponding with this observation, cisplatin treatment induced up-regulation of ER-α36 in a dose-dependent manner in MCF-7, BT474, and MDA-MB-23 cells, respectively (Fig. 1e-h), suggesting that ER-α36 may play an important role during cisplatin resistance formation in breast cancer cells.

**Fig. 1:** Effect of cisplatin on proliferation and ER-α36 expression of breast cancer cells. **a** MCF-7 and MCF-7/DDP cells were treated with increasing concentrations of cisplatin (DDP) for 48 h, and then cell proliferation was measured using CCK-8 assay kit. **b** Cisplatin sensitivity of MCF-7 and MCF-7/DDP cells was examined by monolayer colony formation assay. **c** ER-α36 protein expression in MCF-7 and MCF-7/DDP cells was analyzed using western blot. **d** The quantitative analysis of ER-α36 expression of (**c**). **e** MCF-7 cells were treated with or without 5 μg/mL cisplatin for 48 h, cisplatin-induced expression of ER-α36 was measured by western blot. **f** The quantitative analysis of cisplatin-induced ER-α36 expression of (**e**). **g** MCF-7, BT474 and MDA-MB-231 cells were treated with cisplatin at the indicated concentrations for 48 h and then the protein levels of ER-α36 were analyzed by western blot. **h** The quantitative analysis of cisplatin-induced ER-α36 expression of (**g**). ^*^P < 0.05, ^**^P < 0.01, ^***^P < 0.001

### Overexpression of ER-α36 contributes to cisplatin resistance in breast cancer cells

To explore the potential role of ER-α36 in cisplatin resistance in breast cancer cells, MCF-7 cells stably overexpressing ER-α36 were screened and identified (Fig. 2a and b), and cisplatin sensitivity was detected by cell proliferation and monolayer colony formation assays (Fig. 2c and d). The results revealed that MCF-7/ER-α36 cells obtained resistant phenotype to 5 μg/mL and 10 μg/mL cisplatin, compared with the control cells. Hoechst staining and flow cytometry analysis showed that overexpression of ER-α36 in MCF-7 cells also attenuated cisplatin-induced cell apoptosis (Fig. 2e and f). Collectively, these results suggested that overexpression of ER-α36 contributes to cisplatin resistance in breast cancer cells.

**Fig. 2:** Overexpression of ER-α36 contributes to cisplatin resistance in breast cancer cells. **a** MCF-7 cells stably overexpressing ER-α36 were screened using G418 for 4 weeks and identified by western blot. **b** The quantitative analysis of ER-α36 expression of (**a**). **c** MCF-7/V and MCF-7/ER-α36 cells were treated with increasing concentrations of cisplatin (DDP) for 48 h, and then cell proliferation was measured with CCK-8 assay kit. **d** Cisplatin sensitivity of MCF-7/V and MCF-7/ER-α36 cells was examined by monolayer colony formation assay. **e**, **f** MCF-7/V and MCF-7/ER-α36 cells were treated with or without 5 μg/mL cisplatin for 48 h. The cell nucleus were stained with Hoechst 33258 and then observed under fluorescence microscope. The representative images were shown and the typical apoptotic bodies were marked with white arrows (**e**). The cells were stained with annexin V-FITC/PI. Then the percentage of apoptotic cells was calculated using flow cytometry (**f**). ^*^P < 0.05, ^**^ *P* < 0.01, ^***^P < 0.001

### Knockdown of ER-α36 in cisplatin-resistant breast cancer cells restores cisplatin sensitivity

To further define the significance of ER-α36 in cisplatin resistance, ER-α36 in MCF-7/DDP cells or MCF-7/ER-α36 cells was silenced using siRNA or shRNA and the changes of cell proliferation and monolayer colony formation were analyzed. Western blot analysis showed that transfection of siER-α36 or Lenti-shER-α36 induced a significant knockown of ER-α36 expression compared with the control transfection (Fig. 3a, c, e and g). Cell proliferation assay revealed that cisplatin treatment obviously reduced the proliferation of MCF-7/DDP or MCF-7/ER-α36 cells transfected with siER-α36, compared with the control cells (Fig. 3b and f). Cisplatin treatment significantly decreased monolayer colony number of both MCF-7/DDP cells expressing ER-α36 shRNA and MCF-7/ER-α36 cells expressing ER-α36 shRNA, compared with the control cells (Fig. 3d and h). These data suggested that ER-α36 is an important determinant for cisplatin resistance in breast cancer cells and down-regulation of ER-α36 expression can enhance cisplatin sensitivity.

**Fig. 3:** Knockdown of ER-α36 restores cisplatin sensitivity in cisplatin-resistant breast cancer cells. **a**, **b** MCF-7/DDP cells were transfected with siER-α36 and negative control siRNA (siNC) for 48 h. The cells were collected and analyzed for ER-α36 protein expression using western blot (**a**). The transfected MCF-7/DDP cells were treated with 5 μg/mL cisplatin (DDP) for 48 h, and cell proliferation was measured with CCK-8 assay kit (**b**). **c** ER-α36 expression in MCF-7/DDP cells expressing ER-α36 shRNA and the control cells analyzed using western blot. **d** Cisplatin sensitivity of MCF-7/DDP cells expressing ER-α36 shRNA and the control cells was examined by monolayer colony formation assay. **e**, **f** MCF-7/ER-α36 were treated as in (**a**, **b**), then the peotein level of ER-α36 was detected by western blot (**e**). The proliferation of the transfected MCF-7/ER-α36 cells was evaluated using CCK-8 assay kit (**f**). **g** ER-α36 expression in MCF-7/ER-α36 cells expressing ER-α36 shRNA and the control cells analyzed using western blot. **h** Cisplatin sensitivity of MCF-7/ER-α36 cells expressing ER-α36 shRNA and the control cells was examined by monolayer colony formation assay. ^*^P < 0.05, ^**^P < 0.01, ^***^P < 0.001

### Up-regulation of ER-α36 leads to increased activation of nongenomic estrogen signaling

To clarify the mechanism of ER-α36 involved in cisplatin resistance, we investigated the changes of ER-α36 expression and ER-α36-mediated nongenomic estrogen signaling after cisplatin treatment. In MCF-7 cells, cisplatin treatment induced up-regulated expression of ER-α36 (Fig. 1e-h, 4a, b and d) and activated ER-α36-mediated nongenomic estrogen signaling or the ER-α36/EGFR/HER-2/ERK pathway (Fig. 4a-e). Cisplatin-induced up-regulation of ER-α36 and activation of ER-α36-mediated nongenomic estrogen signaling could also be observed in other breast cancer cell lines including BT474, and MDA-MB-231(Fig. 4d and e). These data suggested that up-regulation of ER-α36 leads to increased activation of nongenomic estrogen signaling. In addtion, cisplatin treatment induced the increased interaction between ER-α36 and EGFR/HER-2 (Fig. 4f), which may further increase the activation of nongenomic estrogen signaling.

**Fig. 4:** Up-regulation of ER-α36 leads to increased activation of nongenomic estrogen signaling. **a** MCF-7 cells were treated with or without 5 μg/mL cisplatin (DDP) for 48 h. Then the protein levels of EGFR, HER-2, ER-α36, total ERK (ERK) and phosphorylated ERK (P-ERK) were detected using western blot. **b**, **c** The quantitative analysis of cisplatin-induced expression of ER-α36, EGFR, HER-2 and P-ERK/ERK of (**a**). **d** MCF-7, BT474 and MDA-MB-231 cells were treated with cisplatin at the indicated concentrations for 48 h and then the protein levels of EGFR, HER-2, ER-α36, ERK and P-ERK were analyzed by western blot. **e** The quantitative analysis of cisplatin-induced expression of P-ERK/ERK of (**d**). **f** MCF-7 cells were treated as in (**a**). The cell lysates were immunoprecipitated with anti-HER-2 or anti-EGFR antibodies. Then the immunoprecipitates were separated by SDS-PAGE and probed with anti-ER-α36 antibodies. Immunoprecipitation of IgG was used as a negative control

### Increased activation of ER-α36-mediated nongenomic estrogen signaling is responsible for cisplatin resistance in breast cancer cells

The previous data have shown that overexpression of ER-α36 in MCF-7/DDP and MCF-7/ER-α36 cells contributes to cisplatin resistance (Figs. 1, 2, 3). Next, we investigated the significance of ER-α36-mediated nongenomic estrogen signaling in cisplatin resistance. Matching with cisplatin-resistant phenotypes of MCF-7/DDP or MCF-7/ER-α36 cells (Figs. 1, 2, 3), the ER-α36/EGFR/HER-2/ERK signaling in these two types of cells was apparently activated compared with the control cells (Fig. 5a and b). However, knockown of ER-α36 in both MCF-7/DDP cells and MCF-7/ER-α36 cells attenuated ER-α36-mediated nongenomic estrogen signaling (Fig. 5c and d), and restored cisplatin sensitivity (Fig. 3). These data suggested that increased activation of ER-α36-mediated nongenomic estrogen signaling is responsible for cisplatin resistance in breast cancer cells.

**Fig. 5:** Increased activation of ER-α36-mediated nongenomic estrogen signaling is responsible for cisplatin resistance. **a**, **b** MCF-7 and MCF-7/DDP cells (**a**) or MCF-7/V and MCF-7/ER-α36 cells (**b**) were harvested and the protein levels of ER-α36, EGFR, HER-2, total ERK (ERK) and phosphorylated ERK (P-ERK) were detected using western blot. **c**, **d** MCF-7/DDP (**c**) and MCF-7/ER-α36 (**d**) cells were transfected with siER-α36 and negative control siRNA (siNC) for 48 h. Then the cells were collected and the levels of ER-α36, EGFR, HER-2, P-ERK, ERK were analyzed by western blot

### Disruption of ER-α36-mediated nongenomic estrogen signaling increases cisplatin sensitivity in breast cancer cells

Since increased activation of ER-α36-mediated nongenomic estrogen signaling is involved in cisplatin resistance in breast cancer cells, we observed whether blocking ER-α36-mediated nongenomic estrogen signaling could increase cisplatin sensitivity in breast cancer cells. Consistent with the previous observation (Fig. 1e-h and Fig. 4a-e), the up-regulation expression of ER-α36 and the activation of ER-α36-mediated nongenomic estrogen signaling in MCF-7 cells were induced again by cisplatin treatment (Fig. 6a). However, cisplatin combined with the EGFR tyrosine kinase inhibitor AG1478 (Sigma-Aldrich, St Louis, MO, USA) or the dual EGFR and HER-2 tyrosine kinase inhibitor Lapatinib (MCE, Monmouth Junction, NJ, USA) or the MAPK/ERK kinase inhibitor U0126 (Sigma-Aldrich, St Louis, MO, USA), significantly inhibited cisplatin-induced expression of ER-α36 and activation of ER-α36-mediated nongenomic estrogen signaling in MCF-7 cells, respectively (Fig. 6a). Meanwhile, the combination of cisplatin and either of the three inhibitors increased cisplatin sensitivity compared with cisplatin treatment alone (Fig. 6b). In cisplatin-resistant MCF-7/ER-α36 cells, the combination of cisplatin and either of the three inhibitors resulted in markedly inhibited phosphorylation of ERK and enhanced cisplatin sensitivity compared with cisplatin treatment alone (Fig. 6c and d). These results suggested that blocking ER-α36 expression or the activity of EGFR/HER-2, or their downstream signaling MAPK/ERK could destroy ER-α36-mediated nongenomic estrogen signaling and thereby increase cisplatin sensitivity in breast cancer cells.

**Fig. 6:** Disruption of ER-α36-mediated nongenomic estrogen signaling increases cisplatin sensitivity in breast cancer cells. **a** MCF-7 cells were treated with or without 5 μg/mL cisplatin (DDP) for 48 h after preincubated with or without AG1478, Lapatinib, and U0126 at the indicated concentrations for 6 h, respectively. Then the levels of ER-α36, total EGFR (EGFR) and phosphorylated EGFR (P-EGFR), total HER-2 (HER-2) and phosphorylated HER-2 (P-HER-2), total ERK (ERK) and phosphorylated ERK (P-ERK) were evaluated using western blot. **b** MCF-7 cells were treated as in (**a**), and then the cell proliferation was measured with CCK-8 assay kit. **c** MCF-7/ER-α36 cells were treated with 5 μg/mL cisplatin for 48 h after preincubated with or without AG1478, Lapatinib, and U0126 at the indicated concentrations for 6 h, respectively. Then the total ERK (ERK) and phosphorylated ERK (P-ERK) was detected by western blot. **d** MCF-7/ER-α36 cells were treated as in (**c**), and then the cell proliferation was examined using CCK-8 assay kit. ^*^P < 0.05, ^**^P < 0.01, ^***^P < 0.001

### Up-regulation of ER-α36 attenuates cisplatin sensitivity in a nude mouse xenograft model

MCF-7/ER-α36 human breast cancer xenografts in Nude Mice were used to evaluate the effect of ER-α36 expression on cisplatin sensitivity in vivo. Cisplatin treatment significantly inhibited the control but not MCF-7/ER-α36 xenograft growth (Fig. 7a and b). ER-α36 expression in MCF-7/ER-α36 xenograft tissues were markedly higher than in control tissues (Fig. 7c), and cisplatin treatment obviously induced up-regulation of ER-α36 in control xenograft tissues (Fig. 7d). These results suggested that up-regulation of ER-α36 can reduce cisplatin sensitivity in vivo.

**Fig. 7:** Up-regulation of ER-α36 attenuates cisplatin sensitivity in a nude mouse xenograft model. **a**, **b** The nude mice bearing MCF-7/V cell-derived and MCF-7/ER-α36 cell-derived subcutaneous tumors were treated intraperitoneally with or without cisplatin (DDP) for 2 weeks, the xenograft tumors were harvested (**a**) and the tumor volume was calculated as described in *Methods* (**b**). **c** ER-α36 protein levels in each group were evaluated by western blot. **d** MCF-7/V tumors treated with or without cisplatin were analyzed for ER-α36 protein levels using western blotting. ^*^P < 0.05, ^**^ *P* < 0.01, ^***^P < 0.001

## Discussion

To the best of our knowledge, this study presents the first evidence that ER-α36 promotes cisplatin resistance in breast cancer cells, which is mediated by increased activation of nongenomic estrogen signaling. Our results suggest that ER-α36 may serve as a novel target to overcome cisplatin resistance as well as a potential biomarker of cisplatin sensitivity in the treatment of breast cancer.

Accumulating evidence has demonstrated that ER-α36 regulates the multiple physiological functions of various tissues. ER-α36 is necessary for ovary development and oocyte meiotic maturation [24] and maintaining the bone density of postmenopausal women [25]. Dysregulation of ER-α36 causes various dysfunctions and diseases, such as osteoporosis, airway hyperresponsiveness, and even cancers [12, 26]. In breast cancer, knockdown of ER-α36 inhibits proliferation, migration, and invasion and increases sensitivity to paclitaxel in MDA-MB-231 cells [27]. ER-α36 also contributes to the proliferation and maintenance of stem-like cells [21, 28]. Specifically, extensive research has shown that ER-α36-mediated nongenomic estrogen signaling is involved in tamoxifen resistance in breast cancer cells [13–15]. In spite of all these investigations, more research is needed to clarify ER-α36 biological function and mechanism. Our current results demonstrated that ER-α36 promotes cisplatin resistance in breast cancer cells, which reveals a new biological function of ER-α36 in the treatment of breast cancer.

The possible mechanism of ER-α36 involved in cisplatin resistance in breast cancer cells was explored in this study. Our current data suggested that ER-α36 promotes cisplatin resistance through nongenomic estrogen signaling. The activation of EGFR/HER-2/ERK signaling is well known cisplatin resistant mechanisms [4, 29, 30]. For example, overexpression of HER-2 leads to the cyclin-dependent kinase inhibitor 1A nuclear exclusion which contributes to cisplatin resistance [4] and it has been related to cisplatin resistance in NSCLC patients [31]. The MAPK/ERK signaling has been associated with both increased and decreased sensitivity to cisplatin in different experiment models [32, 33]. Although the relationship between EGFR/HER-2/ERK signaling and cisplatin resistance in breast cancer cells remains to be defined, the inhibition of the MAPK pathways sensitizes basal-like MDA-MB-468 cells to cisplatin treatment [34]. The high expression of amphiregulin, a specific ligand of the EGFR, shows a highly significant correlation with cisplatin resistance in a variety of human breast cancer cell lines [35]. More importantly, the use of rhuMAb HER-2 in combination with cisplatin in patients with HER-2/neu-overexpressing metastatic breast cancer results in objective clinical response rates higher than those reported previously for cisplatin alone, or rhuMAb HER-2 alone [36]. These studies indicated that activation of EGFR/HER-2/ERK signaling may be involved in cisplatin resistance in breast cancer cells. ER-α36-mediated nongenomic estrogen signaling is characterized by activated EGFR/HER-2/ERK signaling. In our study, we found that cisplatin treatment induced expression of ER-α36 and the interaction between ER-α36 and EGFR/HER-2. Cisplatin-induced up-regulation of ER-α36 enhanced ER-α36-mediated nongenomic estrogen signaling and thereby resulted in cisplatin resistance in breast cancer cells. However, blocking ER-α36 expression or the activity of EGFR/HER-2, or their downstream signaling MAPK/ERK could destroy ER-α36-mediated nongenomic estrogen signaling and thereby increase cisplatin sensitivity. These data suggested that increased activation of ER-α36-mediated nongenomic estrogen signaling is the mechanism of ER-α36 promoting cisplatin resistance in breast cancer cells. Additional, since disruption of ER-α36-mediated nongenomic estrogen signaling could increase cisplatin sensitivity in breast cancer cells, these findings also reveal new therapeutic targets for overcoming cisplatin resistance in breast cancer cells.

Interestingly, both cisplatin-induced expression of ER-α36 and EGFR/HER-2 were observed in our study. It is very important to clarify the potential mechanisms involved in the regulation of ER-α36 and EGFR/HER-2 expression by cisplatin in future. Additional, our current data only demonstrated that cisplatin-induced expression of ER-α36 enhances nongenomic estrogen signaling and confer cisplatin resistance. Considering that there is a regulative relationship between ER-α36 and EGFR/HER-2 [20, 21], it remains unclear whether cisplatin-induced expression of ER-α36 could promote the formation of the ER-α36-EGFR/HER-2 positive regulatory loops and whether these loops may be invovled in cispaltin resistance. The detailed mutual regulatory mechanisms of ER-α36 and EGFR/HER-2 in cispaltin resistance in breast cancer cells need further study.

## Conclusion

In conclusion, our current study demonstrates for the first time that overexpression of ER-α36 promotes cisplatin resistance through nongenomic estrogen signaling. These findings reveal a new important mechanism for the research on cisplatin resistance in breast cancer cells and may provide new strategies to overcome cisplatin resistance by targeting ER-α36. Future research will further explore the significance of ER-α36 expression in breast cancer patients treated with cisplatin.

## Abbreviations

DDP: Cisplatin
EGFR: Epidermal growth factor receptor
ER-α36: Estrogen receptor-alpha36
HER-2: Human epidermal growth factor receptor-2
MAPK: Mitogen-activated protein kinase
ERK: Extracellular signal-regulated kinase
TAM: Tamoxifen
G418: Geneticin
CCK-8: Cell Counting 8 kit
CMV: Cytomegalovirus
Co-IP: Co-immunoprecipitation

## References

[1] Ugur S, Ulu R, Dogukan A, Gurel A, Yigit IP, Gozel N, Aygen B, Ilhan N (2015). The renoprotective effect of curcumin in cisplatin-induced nephrotoxicity. Ren Fail.

[2] Wilmes A, Bielow C, Ranninger C, Bellwon P, Aschauer L, Limonciel A, Chassaigne H, Kristl T, Aiche S, Huber CG, Guillou C, Hewitt P (2015). Mechanism of cisplatin proximal tubule toxicity revealed by integrating transcriptomics, proteomics, metabolomics and biokinetics. Toxicol in Vitro.

[3] Armstrong DK, Bundy B, Wenzel L, Huang HQ, Baergen R, Lele S, Copeland LJ, Walker JL, Burger RA, Gynecologic Oncology G (2006). Intraperitoneal cisplatin and paclitaxel in ovarian cancer. N Engl J Med.

[4] Galluzzi L, Senovilla L, Vitale I, Michels J, Martins I, Kepp O, Castedo M, Kroemer G (2012). Molecular mechanisms of cisplatin resistance. Oncogene.

[5] Shamseddine AI, Farhat FS (2011). Platinum-based compounds for the treatment of metastatic breast cancer. Chemotherapy.

[6] Cohen SM, Lippard SJ (2001). Cisplatin: from DNA damage to cancer chemotherapy. Prog Nucleic Acid Res Mol Biol.

[7] Jamieson ER, Lippard SJ (1999). Structure, recognition, and processing of Cisplatin-DNA adducts. Chem Rev.

[8] Flores-Perez A, Rafaelli LE, Ramirez-Torres N, Arechaga-Ocampo E, Frias S, Sanchez S, Marchat LA, Hidalgo-Miranda A, Quintanar-Jurado V, Rodriguez-Cuevas S, Bautista-Pina V, Carlos-Reyes A (2014). RAD50 targeting impairs DNA damage response and sensitizes human breast cancer cells to cisplatin therapy. Cancer Biol Ther.

[9] Seoane S, Arias E, Sigueiro R, Sendon-Lago J, Martinez-Ordonez A, Castelao E, Eiro N, Garcia-Caballero T, Macia M, Lopez-Lopez R, Maestro M, Vizoso F (2015). Pit-1 inhibits BRCA1 and sensitizes human breast tumors to cisplatin and vitamin D treatment. Oncotarget.

[10] Amable L (2016). Cisplatin resistance and opportunities for precision medicine. Pharmacol Res.

[11] Wang Z, Zhang X, Shen P, Loggie BW, Chang Y, Deuel TF (2005). Identification, cloning, and expression of human estrogen receptor-alpha36, a novel variant of human estrogen receptor-alpha66. Biochem Biophys Res Commun.

[12] Wang ZY, Yin L (2015). Estrogen receptor alpha-36 (ER-alpha36): a new player in human breast cancer. Mol Cell Endocrinol.

[13] Rao J, Jiang X, Wang Y, Chen B (2011). Advances in the understanding of the structure and function of ER-alpha36,a novel variant of human estrogen receptor-alpha. J Steroid Biochem Mol Biol.

[14] Shi L, Dong B, Li Z, Lu Y, Ouyang T, Li J, Wang T, Fan Z, Fan T, Lin B, Wang Z, Xie Y (2009). Expression of ER-{alpha}36, a novel variant of estrogen receptor {alpha}, and resistance to tamoxifen treatment in breast cancer. J Clin Oncol.

[15] Zhang X, Wang ZY (2013). Estrogen receptor-alpha variant, ER-alpha36, is involved in tamoxifen resistance and estrogen hypersensitivity. Endocrinology.

[16] Gu W, Dong N, Wang P, Shi C, Yang J, Wang J (2017). Tamoxifen resistance and metastasis of human breast cancer cells were mediated by the membrane-associated estrogen receptor ER-alpha36 signaling in vitro. Cell Biol Toxicol.

[17] Lin SL, Yan LY, Zhang XT, Yuan J, Li M, Qiao J, Wang ZY, Sun QY (2010). ER-alpha36, a variant of ER-alpha, promotes tamoxifen agonist action in endometrial cancer cells via the MAPK/ERK and PI3K/Akt pathways. PLoS One.

[18] Yin L, Pan X, Zhang XT, Guo YM, Wang ZY, Gong Y, Wang M (2015). Downregulation of ER-alpha36 expression sensitizes HER2 overexpressing breast Cancer Cells to tamoxifen. Am J Cancer Res.

[19] Yin L, Zhang XT, Bian XW, Guo YM, Wang ZY (2014). Disruption of the ER-alpha36-EGFR/HER2 positive regulatory loops restores tamoxifen sensitivity in tamoxifen resistance breast cancer cells. PLoS One.

[20] Zhang XT, Kang LG, Ding L, Vranic S, Gatalica Z, Wang ZY (2011). A positive feedback loop of ER-alpha36/EGFR promotes malignant growth of ER-negative breast cancer cells. Oncogene.

[21] Kang L, Guo Y, Zhang X, Meng J, Wang ZY (2011). A positive cross-regulation of HER2 and ER-alpha36 controls ALDH1 positive breast cancer cells. J Steroid Biochem Mol Biol.

[22] Wang Z, Zhang X, Shen P, Loggie BW, Chang Y, Deuel TF (2006). A variant of estrogen receptor-{alpha}, hER-{alpha}36: transduction of estrogen- and antiestrogen-dependent membrane-initiated mitogenic signaling. Proc Natl Acad Sci U S A.

[23] Chen B, Zhang Y, Wang Y, Rao J, Jiang X, Xu Z (2014). Curcumin inhibits proliferation of breast cancer cells through Nrf2-mediated down-regulation of Fen1 expression. J Steroid Biochem Mol Biol.

[24] Xu BZ, Lin SL, Li M, Zhu JQ, Li S, Ouyang YC, Chen DY, Sun QY (2009). Changes in estrogen receptor-alpha variant (ER-alpha36) expression during mouse ovary development and oocyte meiotic maturation. Histochem Cell Biol.

[25] Xie H, Sun M, Liao XB, Yuan LQ, Sheng ZF, Meng JC, Wang D, Yu ZY, Zhang LY, Zhou HD, Luo XH, Li H (2011). Estrogen receptor alpha36 mediates a bone-sparing effect of 17beta-estrodiol in postmenopausal women. J Bone Miner Res.

[26] Su X, Xu X, Li G, Lin B, Cao J, Teng L (2014). ER-alpha36: a novel biomarker and potential therapeutic target in breast cancer. Onco Targets Ther.

[27] Zhang J, Li G, Li Z, Yu X, Zheng Y, Jin K, Wang H, Gong Y, Sun X, Teng X, Cao J, Teng L (2012). Estrogen-independent effects of ER-alpha36 in ER-negative breast cancer. Steroids.

[28] Deng H, Zhang XT, Wang ML, Zheng HY, Liu LJ, Wang ZY (2014). ER-alpha36-mediated rapid estrogen signaling positively regulates ER-positive breast cancer stem/progenitor cells. PLoS One.

[29] Muller CB, De Bastiani MA, Becker M, Franca FS, Branco MA, Castro MA, Klamt F (2015). Potential crosstalk between cofilin-1 and EGFR pathways in cisplatin resistance of non-small-cell lung cancer. Oncotarget.

[30] Pietras RJ, Fendly BM, Chazin VR, Pegram MD, Howell SB, Slamon DJ (1994). Antibody to HER-2/neu receptor blocks DNA repair after cisplatin in human breast and ovarian cancer cells. Oncogene.

[31] Citri A, Yarden Y (2006). EGF-ERBB signalling: towards the systems level. Nat Rev Mol Cell Biol.

[32] Persons DL, Yazlovitskaya EM, Pelling JC (2000). Effect of extracellular signal-regulated kinase on p53 accumulation in response to cisplatin. J Biol Chem.

[33] Yeh PY, Chuang SE, Yeh KH, Song YC, Ea CK, Cheng AL (2002). Increase of the resistance of human cervical carcinoma cells to cisplatin by inhibition of the MEK to ERK signaling pathway partly via enhancement of anticancer drug-induced NF kappa B activation. Biochem Pharmacol.

[34] Wong SW, Tiong KH, Kong WY, Yue YC, Chua CH, Lim JY, Lee CY, Quah SI, Fow C, Chung C, So I, Tan BS (2011). Rapamycin synergizes cisplatin sensitivity in basal-like breast cancer cells through up-regulation of p73. Breast Cancer Res Treat.

[35] Eckstein N, Servan K, Girard L, Cai D, von Jonquieres G, Jaehde U, Kassack MU, Gazdar AF, Minna JD, Royer HD (2008). Epidermal growth factor receptor pathway analysis identifies amphiregulin as a key factor for cisplatin resistance of human breast cancer cells. J Biol Chem.

[36] Pegram MD, Lipton A, Hayes DF, Weber BL, Baselga JM, Tripathy D, Baly D, Baughman SA, Twaddell T, Glaspy JA, Slamon DJ (1998). Phase II study of receptor-enhanced chemosensitivity using recombinant humanized anti-p185HER2/neu monoclonal antibody plus cisplatin in patients with HER2/neu-overexpressing metastatic breast cancer refractory to chemotherapy treatment. J Clin Oncol.

